The article "The Application of Transcranial Electrical Stimulation in Sports Psychology" was published in 2022. Journal: Comput Math Methods Med.

# The Application of Transcranial Electrical Stimulation in Sports Psychology

**DOI:** 10.1155/2022/1008346

**Published:** 2022-07-13

**Authors:** Shuzhi Chang

**Affiliations:** ^1^Teaching Laboratory and Training Center, Tianjin University of Sport, Tianjin 301617, China; ^2^Key Laboratory of Competitive Psychological and Physiological Regulation of General Administration of Sport, Tianjin University of Sport, Tianjin 301617, China

## Abstract

The problem of sports psychological fatigue has become one of the focal points of common concern among scholars at home and abroad. Athletes will face many problems and challenges in competition or training, and if they are not handled properly, they will have negative experiences, which will affect the training benefits and develop psychological fatigue. Transcranial electrical stimulation (TES), which contains transcranial direct current stimulation, transcranial alternating current stimulation, and transcranial random noise stimulation, is a noninvasive brain stimulation method. By applying specific patterns of low-intensity electrical currents to specific brain regions through electrodes of different sizes, it modulates cortical neural activity and/or excitability and enhances the connections between the brain and nerves and muscles to achieve improved motor performance. TES technology is currently making the transition from laboratory research to applied research in sports science. In this paper, we first describe the neural mechanisms of TES action on the cerebral cortex, including five aspects of body balance, endurance performance, exercise fatigue, muscle strength, and motor learning ability; then, we review the relevant studies on the application of TES in functional connectivity of brain networks and explore the importance of this field for TES to improve athletic performance. This research provides a machine learning-based and transcranial electrical stimulation model for the locomotor psychological fatigue problem in rock climbers since rock climbing is a sport that places great demands on athletes' psychological quality. The research on the factors influencing the psychological fatigue of climbers and the intervention measures is beneficial to the early diagnosis and the prevention and intervention of it.

## 1. Introduction

In modern high water competitive sports, the physical and technical and tactical abilities of the participating athletes are getting closer and closer, and the stable psychological quality becomes an important factor to achieve the victory of the competition, especially the climbing sports competition has a greater consumption of the athletes' psychological energy; if the athletes do not have good psychological quality, even if they have strong physical quality, technical, and tactical ability, it is difficult to achieve excellent sports performance. As the American scholar Grubaugh pointed out for junior athletes, 80% is biomechanical factors, 20% is psychological factors, senior athletes are the opposite, 80% is psychological factors, and 20% is biomechanical factors. Therefore, in the process of physical and technical and tactical training for rock climbers, it is crucial to strengthen the psychological quality training of athletes.

In rock climbing sport characteristics and climbing psychological training, climbing site, and the sport form of special, climbing site mainly rock cliff face fissure rock face boulder and artificial rock wall, etc., the rock face mostly has a certain elevation angle and pitch angle, and the shape of the rock wall and rock point of the shape of a thousand changes, thus forming the form of rock-climbing sport diversity unconventional work at height and the complexity of technical operations and other characteristics [1–3].  Figure 1 depicts the diagram for using rock climbing to enhance psychological quality. A set of difficult and beautiful sports, rock climbing is demanding and risky. Its core traits can be summed up as dangerous, difficult, and beautiful. The angle and shape of the rock wall, the difficulty of the climbing route, the size and shape of the pivot points, and the ever-changing weather are all huge obstacles to climbing; so, athletes are required to have strong resilience and adjust their physical and mental state to better complete the competition. If you make a mistake, you may have the danger of slipping and falling, and you are prone to casualties. Rock-climbing psychological training refers to the process of rock-climbing training, purposely and systematically exerts influence on the psychological process and personality psychological characteristics of athletes, and through special methods and means to make athletes learn to regulate and control their own psychological state, and then regulates and controls their own climbing behavior process due to the specificity of the rock-climbing site the variability of the wall pivot points the diversity of equipment preparation the complexity of technical actions, and it can promote the perfection of athletes' psychological process, form good personality and psychological characteristics compatible with rock climbing, obtain a high level of psychological energy reserves, enable athletes to adapt to the thrilling climbing activities, and lay a good psychological foundation for the victory of the climbing competition. The climbing competition is carried out under the condition of independent combat without guidance, and in the application of techniques and tactics in the process of the competition, the athletes should make timely self-adjustment according to the difficulty angle of the line pivot point and personal advantages and disadvantages of the competition. Good psychological quality makes athletes confident of victory, energetic, vigorous, muscular strength, and increased resilience, so that they can give full play to their existing skills and tactics, and even play beyond the level of psychological training is generally divided into psychological training and psychological training in preparation for specific competitions. General psychological training aims to improve the psychological factors of athletes related to special sports and is also called long-term psychological training because it can be arranged throughout the training process. Psychological training in preparation for specific competitions is mainly for the specific competition and psychological preparation, generally in the two or three months before the competition to start practicing, and continues until the competition period pregame special psychological training aims to enable athletes to master and use the method of self-regulation of mental state in a relatively short period of time, in order to form the best competitive state [4–6].

Human motor control ability is one of the important motor abilities of the human body. Motor control not only affects the athletes' performance but also has a significant impact on the quality of life of healthy people in general, especially the elderly and patients with motor control deficits. Previous approaches to improve motor control in humans have focused on enhancing motor control through interventional training to modify the function of the skeletal muscle system. However, the nervous system plays a very important role in the process of motor control. In recent years, research on motor control has focused more on the effects of neurological interventions on human motor control [7]. Transcranial electrical stimulation (TES) is a noninvasive transcranial electrical stimulation technique that generates a weak current (1 to 2 mA) in the superficial layers of the skull through paired electrodes placed on the scalp, which affects neural activity in the cerebral cortex and alters brain function to promote motor performance in humans. The main transcranial electrical stimulation techniques used today are transcranial direct current stimulation (tDCS), transcranial alternating current stimulation (tACS), and transcranial random noise stimulation (TRS). These electrical stimulation techniques can be used to achieve different stimulation effects by changing the position of electrodes, the intensity of current, the duration of stimulation, and the frequency of stimulation. As a noninvasive and safe brain stimulation technique, TES has been gradually announced into sports science applications from the treatment of neurological or psychiatric disorders. In this paper, we focus on the research and application of TES in improving sports mental performance, especially in rock climbing. A machine learning algorithm-based transcranial electrical stimulation in sports psychology is proposed for applications including improving mental balance, enhancing mental endurance performance and/or relieving exercise fatigue, improving muscle strength, and enhancing sports psychological learning ability, which provides theoretical references for better understanding and application of TES techniques. The effectiveness of the proposed method was demonstrated in relevant experiments [8].

The usefulness of transcranial electrical stimulation in enhancing psychomotor balance, psychomotor endurance performance, psychomotor strength, and decreasing motor fatigue is further examined in this paper.

The arrangements of the paper are as follows: Section 2 discusses the related work.  Section 3 examines the various methods.  Section 4 analyzes the experiments and results.  Section 5 concludes the article.

## 2. Related Work

### 2.1. Transcranial Electrical Stimulation and Sports

Currently, TES is more frequently used in the rehabilitation of patients with neurological impairment or psychiatric disorders and has good belongings on the recovery of brain injury, mood regulation, and improvement of cognitive function. In recent years, some researchers have gradually applied TES to the field of sports science to improve human muscle coordination in sports and enhance human sports performance by increasing the connection between the brain and nerves and muscles, such as improving body balance, enhancing endurance performance, relieving sports fatigue, and improving muscle strength and motor learning ability. Improve body balance ability is one of the main physical qualities of humans, which refers to the ability to maintain body posture even during exercise or under external forces, and it is related to body structure, muscle coordination, and the regulation of brain tissue involved in balance [9–12]. It was found that 1 mA tDCS anodal stimulation of the motor cortex of healthy elderly people for 20 min per day resulted in improved gait and dynamic balance after 5 d of continuous intervention and was maintained for 1 week. Stimulation of the sensorimotor area of healthy adults with high precision tDCS for 20 min better the static balance ability of the subjects. Body balance is one of the basic abilities that athletes possess, especially in nonperiodic events, and directly affects the performance of athletes' skills and physical abilities, etc. Whether tDCS can improve dynamic and static balance in elite athletes needs further study. Enhance endurance performance and/or relieve exercise and fatigue. Endurance is the body's ability to perform muscle activity for long periods of time and is the basis for improving qualities such as speed and strength. The goodness of endurance directly affects human athletic performance. Currently, some studies have investigated whether tDCS intervention in the cerebral cortex has a positive effect on neurological and muscular fatigue recovery [13].

The exact neurophysiological mechanisms of transcranial direct current action can be divided into the following mainstream views: altering cortical excitability, increasing synaptic plasticity, altering local cerebral blood flow, and regulating local cortical and brain network connections. Changing cortical excitability is as follows: tDCS changes the excitability of the brain by stimulating the membrane potential of neurons, causing depolarization of the anode to lower the threshold of action potential generation, and increasing the excitability of the anodal cortex; [14–16]. Increase synaptic plasticity is as follows: tDCS performs subthreshold stimulation of the resting membrane potential of neurons, which induces the expression of N-methyl aspartate receptors and the release of y-aminobutyric acid, while NMDA is involved in synapse formation, increasing synaptic plasticity, which in turn produces long-duration inhibitory or enhancing effects. Alteration of local cerebral blood flow is as follows: when the tDCS anode acts on the dorsolateral prefrontal cortex, it increases cerebral blood flow in the stimulated area and decreases cerebral blood flow under the cathode, which is highly correlated with the MEP amplitude at the stimulation location. Modulation of local cortical and brain network connectivity is as follows: EEG and functional magnetic resonance imaging studies revealed that anodal tDCS stimulation of area M1 significantly increased functional connectivity in the premotor, motor, and sensorimotor areas within the stimulated hemisphere and induced changes in connectivity between the left and right hemispheres, further corroborating that tDCS induces functional brain connectivity. tACS stimulation is dependent on the stimulation. The mechanisms of tACS action can be classified as follows: exogenous oscillations induce endogenous oscillations in the brain, affecting synaptic plasticity to regulate brain function. When tACS acts on the brain, part of the current reaches the cerebral cortex and changes the membrane potential of dendrites or axons in an oscillatory manner, making it possible for neurons to develop action potentials. When the frequency of tACS is the same as the endogenous frequency, resonance occurs, causing excitation of neurons in the brain; when tACS is stimulated at a higher frequency, it can trigger neuronal oscillations in a wider frequency range. Stimulation at specific frequencies can also drive oscillatory frequencies within the brain and induce synchronous oscillations in neurons with rhythms imposed by tACS on specific cortices. tACS modulates brain function by affecting synaptic plasticity. When tACS causes presynaptic action potentials to precede postsynaptic action potentials, it produces long-lasting excitation of brain function, and when it causes postsynaptic potentials to precede presynaptic potentials, it causes long-lasting inhibition of brain function, a phenomenon that has been confirmed by many studies.

### 2.2. Psychological Analysis of Rock Climbing

Rock climbing is a kind of mountaineering sport, which fully exploits the human body's climbing potential, and the climber relies on the coordination of hands, feet, waist, and muscle functions and uses gouging, grasping, bracing, and other means to operate the body upward. Both man-made and natural rock walls can be climbed, with man-made rock walls having the most participants. According to the psychological requirements of rock climbing, climbers must perform well in specialized psychological quality training to improve their capacity for psychological adjustment and obstacle surmounting [17–19]. The sport of rock climbing demands exceptional physical, intellectual, and psychological qualities.

Rock climbing is a sport with long time, high density, and large volume of transportation. The process of rock climbing puts forward extremely high requirements on athletes' physical ability, and athletes need strong physical ability, intelligence, and good psychological quality to complete a complete climb. In the process of rock climbing, the athletes' psychological ability is extremely important. In the process of rock climbing, due to the rapid consumption of physical energy, it often causes a rapid decline in the athletes' functional reserve and central nervous fatigue, which leads to a series of bad emotions such as inattention, irritability, and decrease in the level of will. If these bad emotions deteriorate further, it will cause the athletes to move slowly, have stiff muscles, and panic in their hands and feet. These bad emotions, if further worsened, will cause the athletes to move slowly, muscle stiffness, and hands and feet panic, affecting the completion of rock climbing. In serious cases, it will lead to sports injury or even danger. Therefore, the special psychological training for rock climbers is extremely important, through effective psychological training, so that athletes can effectively psychologically regulate themselves in the process of rock climbing and help them maintain emotional stability [20, 21]. We know that rock climbing has a certain degree of danger, and the psychology of fear in the procedure of rock climbing is caused by a variety of reasons. One of the most important factors is the climber's understanding of the degree of obstacles and the climber's level of trust in protective events and protection personnel. To train and improve climbers to overcome psychological barriers, it is necessary to find the cause and prescribe the right remedy: first, to make climbers fully understand the degree of difficulty of this climb and some related knowledge and second, to make climbers do good communication with staff to enhance their trust in protection workers and safety measures.

Concentration training is extremely important for rock climbers. Only by concentrating on one goal can the climber not be disturbed by the external environment and internal factors during the climbing process, not be distracted during the climbing, and reach the summit successfully. The concentration of attention training generally has two forms: one is the muzzle training method: the so-called muzzle training refers to the trainer in the usual training by issuing some volume weak, just can barely hear the sound, and let the trainee to complete the task, and such a weak voice muzzle needs athletes to focus on a high degree of attention to complete. Second is the stopwatch training method [22]. The so-called stopwatch training is to allow athletes to focus on the rotation of the stopwatch, record the time of each attentiveness, in the training time lengthened one by one, until the end of inattention, and then repeat the training in accordance with this time standard. Training regulates arousal level in rock climbing; there are two kinds of training to regulate arousal level in rock climbing: one is to increase the arousal level of AH, and the other is to decrease, the arousal level of sex. Arousal level refers to the physiological activation of the muscles in different degrees and states, and the state of arousal level is directly related to the level of athletes. The human body can change and maintain the excitability of the brain's nervous system through arousal and use this state of arousal to maintain a high level of concentration and provide conscious energy to the muscles. In general, in sports that are mainly speed and strength-based, a higher level of arousal is required, while in sports that are mainly regulated by small muscle groups and have complex tasks. Exercise classes that require coordinated coordination require a lower level of arousal [23].

The so-called representational training refers to the training to promote the athletes to improve their climbing skills and technical level of play; in the representational training, coaches can make the athletes form the representational movement in the brain consciousness through verbal explanation, video images, video materials, and other means, so that the athletes can train through the full imagination. The main purpose of representational training is to allow athletes to train in actual combat before. In addition, representational movement also includes the reproduction of previously learned technical movements after training, through the recollection and reproduction of movements in the brain, the wrong movements can be corrected, and the correct movements can be consolidated. In the process of representational training, athletes can categorize and organize the decomposed movements one by one in their mind and make corrections and improvements, so that they can complete the whole climbing process independently in their own mind. Representation training not only makes the athletes get twice the result with half the effort in the climbing process but also increases the information reserve and develops their intelligence.

## 3. Methods

### 3.1. Model Architecture

Decoding and analyzing the event-related desynchronization/event-related synchronization generated by the conceptual activity of rock climbing to determine the user's motor intention and brain state are the basis for the implementation of a brain-machine interface based on the psychology of rock-climbing. Users gain the ability to actively regulate their sensorimotor rhythms to give control commands in the psychological brain-machine interface based on rock climbing. The modulation patterns induced by psychomotor rhythms in the brain can be used as control input signals for the BCI, and through learning and training, climbers can autonomously generate the corresponding EEG patterns. The model structure diagram of the psycho-brain-computer interface for rock climbing is shown in Figure 2. The system is similar to other brain-computer interface systems and is generally composed of the following parts: signal acquisition part, signal preprocessing, feature extraction, pattern classification, and output module. Signal acquisition part is as follows: the main role is to record the EEG signals that the subjects go through the psychological experiment paradigm of rock-climbing exercise and thus generate. Signal preprocessing is as follows: the preprocessing stage is mainly to remove the noise from the EEG signal, usually using a band-pass filter, and to remove the electrooculography and motion artifacts using various methods as needed. Feature extraction is as follows: since the EEG signals of climbers during the mental activity of rock-climbing sports are mixed with those generated by other neural activities and are overwhelmed by a large amount of spontaneous EEG, the feature signals related to the mental activity of rock-climbing sports need to be extracted from these mixed EEG signals by reducing the dimensionality of the EEG signals so as to extract the relevant features. Pattern classification is as follows: the extracted to feature information is analyzed and judged, so that these features can be decoded into various instructions or parsed into the user's intention of rock-climbing sports psychology. Output module includes two parts: control system and feedback system. There are some brain-machine interfaces based on rock-climbing psychology aiming at helping paralyzed climbers to perform some daily activities, and then the extracted feature information will be decoded into various control commands to control external devices, such as robots, wheelchairs, and mice. There are also some brain-machine interfaces based on the psychology of rock climbing, whose purpose is to help climbers with neurological damage to carry out neural pathway rehabilitation or healthy climbers to improve their athletic ability through the psychological training of rock-climbing, without controlling external devices, and then the decoded commands will be analyzed and returned to the climbers through the feedback system.

### 3.2. Preprocessing

In this paper, after the EEG data are acquired, the calculation of subject-specific band *r*^2^ is performed in the preprocessing stage for the determination of the subject's band-pass filter. *r*^2^ is calculated as follows.

(1) $$\begin{array}{c} r^{2}={\left(\frac{\sqrt{N_{1}N_{2}}}{N_{1}+N_{2}}\frac{\text{MEAN}\left(P_{1}\right)-\text{MEAN}\left(P_{2}\right)}{\text{STD}\left(P_{1}\cup P_{2}\right)}\right)}^{2}. \end{array}$$

In the equation, *N*_1_ and *N*_2_ are the number of tasks included in the EEG data, respectively, *N*_1_ represents the number of trails for the left-hand motor imagery task, and *N*_2_ represents the number of trails for the left-hand motor imagery task. *P*_1_ and *P*_2_ are the power spectra of the EEG data for the motor imagery task, *P*_1_ represents the power spectrum of the left-hand motor imagery EEG data, and *P*_2_ represents the power spectrum of the right-hand motor imagery EEG data. The larger the value of *r*^2^, the greater the energy difference between the EEG data of left- and right-handed motor imagery tasks in that frequency band. According to the value of *r*^2^, a suitable band-pass filtering band is selected to perform specific band-pass filtering on the motor imagery EEG data, followed by CSP feature extraction and LDA pattern classification.

### 3.3. Feature Extraction

The flow of signal data feature extraction is shown in Figure 3. For the together EEG signals, there are three main features: time domain features, frequency domain features, and spatial domain features, and we need to choose the corresponding feature extraction methods for dissimilar features. For example, spatial domain features are usually extracted by choosing spatial domain filters—Common Spatial Pattern (CSP), while frequency domain features are generally extracted by power spectrum analysis and some other wavelets transform, sample entropy method, etc. Each of these methods has its own advantages and disadvantages, as shown in Table 1.

In this study, the purpose is to extract the two characteristic signals of left-handed motion and right-handed motion generated by the user's motion imagination, and using the CSP algorithm is more in line with our requirements. The CSP algorithm is to calculate all channels, and we know that the variance represents the energy, due to the phenomenon of ERD/ERS generated by motion imagination, and it is easier to use the CSP algorithm. Because of the ERD/ERS phenomenon, it is easier to extract the features with the greatest difference in energy to classify the motor imagery intention.

### 3.4. CSP Algorithm

The CSP algorithm is a feature extraction algorithm for two arrangement tasks. The computational procedure of the CSP algorithm is as follows: assume that *X*_1_ and *X*_2_ are the matrices of the single evoked EEG signals under the same experimental conditions of the left and right handed two motor imagery responsibilities, respectively, and the matrix dimension *N*^∗^*T*, *N* is the number of channels of EEG signals, and *T* is the number of sampling points of EEG signals, as the number of channels of EEG signals commonly used is 8 conductors, 16 conductors, 32 conductors, 64 conductors, and 128 conductors. *N* must be less than *T* to satisfy the condition of calculating the covariance matrix. Specify that *Y*_1_ and *Y*_2_ are two types of tasks for left-handed motion and right-handed motion, and *X*_1_ and *X*_2_ are represented as follows, respectively, when noise interference is ignored.

(2) $$\begin{array}{c} X_{1}=\left[A_{1}A_{m}\right]\left[\begin{array}{c} Y_{1}\\ Y_{M} \end{array}\right],X_{2}=\left[A_{2}A_{m}\right]\left[\begin{array}{c} Y_{2}\\ Y_{M} \end{array}\right]. \end{array}$$

Assume that the source signals of the two tasks, *Y*_1_ for left-handed motion and *Y*_2_ for right-handed motion, are linearly independent of each other, *Y*_*u*_ represents the common source signal possessed by these two tasks, *Y*_1_ consisting of *m*_1_ sources and *Y*_2_ consisting of *m*_2_ sources, then *A*_1_ consists of *m*_1_ covariance patterns associated with *X*_1_, *A*_2_ consists of *m*_2_ covariance patterns associated with *X*_2_. The purpose of the CSP algorithm is to design a spatial filter parameter to obtain the best projection matrix *W*. The EEG signals are passed through this spatial filter to obtain new signals where one has the largest variance, the other has the smallest variance, and then the two types of signals are classified by a classification algorithm. Calculate the covariance matrix of *X*_1_ and *X*_2_, respectively.

(3) $$\begin{array}{c} \begin{array}{c} R_{1}=\frac{{X_{1}X_{1}}^{T}}{\text{tr}\left(X_{1}X_{1}^{T}\right)},\\ R_{2}=\frac{X_{2}X_{2}^{T}}{\text{tr}\left(X_{2}X_{2}^{T}\right)}, \end{array} \end{array}$$

*r* denotes the trace of the matrix, which is the sum of the diagonal elements of the matrix *X*_1_*X*_1_^*T*^. Here, *R*_1_ and *R*_2_ are the covariance matrices for a single trial, and then the respective average covariance matrices *R*_1_ and *R*_2_ are calculated based on the total number of trials for each of the left- and right-hand tasks, denoted as *n*_1_ and *n*_2_:

(4) $$\begin{array}{c} \begin{array}{c} \overset{¯}{R_{1}}=\frac{1}{n_{1}}\overset{n_{1}}{\underset{i=1}{\sum }}\;R_{1i},\\ \overset{¯}{R_{2}}=\frac{1}{n_{2}}\overset{n_{2}}{\underset{i=1}{\sum }}\;R_{2i}. \end{array} \end{array}$$

Calculate the mixed-space covariance matrix *R*.

(5) $$\begin{array}{c} R=\overset{¯}{R_{1}}+\overset{¯}{R_{2}}. \end{array}$$

Since the obtained mixed-space covariance matrix *R* is a positive definite matrix, the eigenvalue decomposition of the obtained mixed-space covariance matrix *R* is performed according to the singular value theorem as follows.

(6) $$\begin{array}{c} R=U\lambda U^{T}. \end{array}$$

*λ* denotes the diagonal matrix composed of eigenvalues arranged in descending order, and *U* denotes the matrix composed of eigenvectors corresponding to the decomposed eigenvalues, resulting in the whitening transformation matrix *P*.

(7) $$\begin{array}{c} P=\frac{1}{\sqrt{\lambda U^{T}}}. \end{array}$$

For the formal experimental data, to avoid transient abrupt changes in the EEG signal caused by body movements, its variance is calculated and normalized for the eigensignal obtained through the spatial filter, and then the eigenvectors are extracted as follows.

(8) $$\begin{array}{c} \left\{\begin{array}{c} Z_{i}=WX_{i},\\ f_{i}=\frac{\mathrm{var}\left(Z_{i}\right)}{\sum \mathrm{var}\left(Z_{i}\right)}. \end{array}\right. \end{array}$$

### 3.5. Pattern Classification

To interpret the subject's motor imagery intention and to differentiate the brain activity caused by left-handed and right-handed motor imagery activities, the recovered features from the EEG signal must be sent to a classifier for pattern classification after the signal has been retrieved. The algorithms used to categorize the extracted features into patterns are both linear and nonlinear, and the linear algorithms include linear discriminant classifiers and linear classifiers of Marxian distance, among others. Based on the above mentioned and the characteristics of motor imagery EEG signals.

LDA is an effective feature extraction method that can classify data and compress the feature space dimension. This section introduces the basic principle of LDA starting from the simpler class II LDA. First assume that there are *m* samples in the dataset, denoted as

(9) $$\begin{array}{c} D=\left\{\left(x_{1},y_{1}\right),\left(x_{2},y_{2}\right),\cdots ,\left(x_{m},y_{m}\right)\right\}, \end{array}$$

where *x* is an *n*-dimensional vector and *y*_*i*_ ∈ {0, 1}. We define *N*_*j*_(*j* ∈ {0, 1}) as the number of samples of the *j*-th class and *N*_*j*_(*j* ∈ {0, 1}) as the set of samples of the *j*-th class, and then the mean vector of samples of the *j*-th class can be expressed as

(10) $$\begin{array}{c} \mu_{j}=\frac{1}{N_{j}}\underset{x\in X_{j}}{\sum }\;x,j\in \left\{0,1\right\}. \end{array}$$

The covariance matrix of the *j*-th class of samples can be expressed as

(11) $$\begin{array}{c} \Sigma_{j}=\underset{x\in X_{j}}{\sum }\;\left(x-\mu_{j}\right){\left(x-\mu_{j}\right)}^{T},j\in \left\{0,1\right\}. \end{array}$$

The projection vector is denoted by *w*. Then, any sample *x* becomes *w*^*T*^*x*_*i*_ after projection. As mentioned above, the purpose of the LDA algorithm is to make the distance between similar data as small as possible, and the distance between different classes of data as large as possible.

(12) $$\begin{array}{c} G_{1}=w^{T}\Sigma_{0}w+w^{T}\Sigma_{1}w. \end{array}$$

The distance between samples of different categories is expressed as the square of the second parametric number, as follows:

(13) $$\begin{array}{c} G_{2}={||w^{T}\mu_{0}-w^{T}\mu_{1}||}_{2}^{2}. \end{array}$$

In summary, the optimization objective of the LDA algorithm is

(14) $$\begin{array}{c} w^{*}=\underset{w}{\arg\max}\frac{G_{2}}{G_{1}}=\frac{{||w^{T}\mu_{0}-w^{T}\mu_{1}||}_{2}^{2}}{w^{T}\Sigma_{0}w+w^{T}\Sigma_{1}w}=\frac{w^{T}\left(\mu_{0}-\mu_{1}\right){\left(\mu_{0}-\mu_{1}\right)}^{T}w}{w^{T}\left(\Sigma_{0}+\Sigma_{1}\right)w}. \end{array}$$

## 4. Experiments and Results

In this section, it discusses the various experimental setups and define the transcranial electrical stimulation. They analyze the experimental results.

### 4.1. Experimental Setup

This chapter investigates the effects of transcranial electrical stimulation on motor imagery task ability based on the motor imagery brain-machine interface. In the ERD/ERS data, changes in classification accuracy before and after transcranial electrical stimulation were analyzed separately to investigate the electrophysiological effects of transcranial electrical stimulation on motor imagery. This experiment was a single-blind experiment, subjects were required to perform a total of four experiments, and the sequence of stimulation and control experiments was randomly arranged by the main subjects. To avoid the after-effects of transcranial electrical stimulation, the time interval between each group of stimulation and control experiments was ensured to be at least 24 hours.

Ten rock climbers (age range 23-25 years, mean age 24.4 ± 0.44 years) were recruited for this experiment, and all participants were active climbers and received monetary compensation. During the experiment, subjects would receive a total of four MI task experiments and three transcranial electrical stimulations. The subjects first underwent the first MI task experiment to determine the baseline level of each outcome for comparison and analysis with the subsequent experiments, followed by three randomized transcranial electrical stimulation sessions with corresponding MI task experiments and EEG recordings. The duration of the after-effects of transcranial direct current stimulation is not more than 10 min, and the duration of the after-effects of transcranial alternating current stimulation has not been systematically studied, but the duration of the after-effects of 10 Hz, 1 mA alternating current stimulation, is 30 min; so, the interval between each stimulation is guaranteed to be more than 24 h to avoid the after-effects from affecting the results of the subsequent experiments. The experimental parameters are set as shown in Table 2.

### 4.2. Transcranial Electrical Stimulation

1. Electrical stimulation equipment: publicly available transcranial electrical stimulation equipment. It is capable of three stimulation modes tACS, and pseudostimulation
2. Stimulation intensity: (a) tDCS: all subjects uniformly use 1 mA current intensity, and the stimulating electrodes use 5^∗^7 cm saline soaked sponge electrodes. (b) tACS: The stimulation intensity was determined according to the subject's stimulation threshold specificity as described, and the stimulation electrode was a 5^∗^7 cm saline-soaked sponge electrode
3. Stimulation position: the electrode placement was as shown in Figure 4, with the anode placed at the location of the motor sensory M1 area and the cathode electrode located at the forehead area
4. Stimulation frequency: 10 Hz (mean of *μ* rhythm) was used to stimulate the subjects during the tACS experiment. (5) Stimulation time: for both tACS and tDCS, a current stimulation lasting 10 min was applied to the subjects

After the raw EEG data were collected and pre-processed, the LDA algorithm was used to calculate the classification accuracy of the EEG data for the two motor imagery tasks, as well as to calculate the power spectrum of the EEG data in the prestimulation and poststimulation phases to observe the changes in ERD/ERS, respectively. The diagram of the training process performance improvement is shown in Figure 5.

### 4.3. Experimental Results

For motor mental classification accuracy, this paper used one-way frequent measures ANOVA to test the significance of the classification accuracy of subjects' motor imagery before and after different experimental conditions. *p* < 0.05 was considered to be a significant difference. Among the ten subjects, one subject's data was eliminated for excessive noise, and the EEG data of the remaining nine subjects were finally used for the analysis. The accuracy of subjects' psychological recovery during rock climbing exercise is shown in Table 3.

The average accuracy of task classification is shown in Figure 6. A one-way repeated measures ANOVA was performed on the four experimental groups, *F* (3, 24) = 10.436, *p* < 0.05, indicating a significant main effect. The following results were obtained from a two-by-two comparison of the four experimental groups: tACS group compared to tDCS compared to the prestimulus group experiment, *p*_1_ = 0.08 > 0.05 and *p*_2_ = 0.002 < 0.05, respectively, and tACS group compared to tDCS compared to the pseudostimulus group experiment, *p*_3_ = 0.193 > 0.05 and *p*_4_ = 0.02 < 0.05, respectively. From the classification accuracy of the MI task in the four groups, it can be seen that the accuracy of the subjects after the tDCS inspiration was significantly improved compared to the prestimulation and pseudostimulation groups, and the accuracy of the subjects after the tACS stimulation was better quality compared to the prestimulation and pseudostimulation groups but was not significant. In terms of the overall level of accuracy improvement, tDCS was more effective in improving classification accuracy than the tACS group.

The visualization results of the accuracy of mental recovery in rock climbing without and with transcranial electrical stimulation are shown in Figures 7 and 8, respectively. From the individual subjects' point of view, the accuracy of motor imagery was effectively improved in all nine subjects after tDCS stimulation. For tACS, subjects 5 and 8 showed a decrease in accuracy after tACS compared to the prestimulation period, and subjects 1, 3, and 6 showed a better increase in accuracy after tACS than they did after tDCS. Among all the subjects in the experimental group, the highest accuracy rate was that of subject 1 after tACS inspiration, with an accuracy rate of 98.75%. Among all subjects in the experimental group, the lowest accuracy rate was for subject 8 after tACS stimulation, with an accuracy rate of 75.11%.

## 5. Conclusion

Rock climbing requires climbers to have good psychological quality, and these psychological qualities include the ability to overcome anxiety, fear, and obstacles, but also includes the level of the athlete's will, the degree of concentration, etc. The psychological training of climbers should be targeted according to the specific characteristics of each athlete to improve their psychological mechanisms through training.

The brain controls most of the human learning and movement. Although sports training focuses on physical performance and motor abilities, its fundamental nature still depends on the cerebral cortex to create neural connections that help the nervous system better govern muscles. There is a transcranial electrical stimulation's efficiency in enhancing human motor performance. This paper further analyzes the effectiveness of transcranial electrical stimulation in improving psychomotor balance, psychomotor endurance performance, and psychomotor strength and reducing motor fatigue.

## Figures and Tables

**Figure 1:** Rock climbing to enhance the psychological quality of the schematic diagram.

**Figure 2:** Model structure.

**Figure 3:** Signal data feature extraction process.

**Figure 4:** Stimulation electrode location map.

**Figure 5:** Schematic diagram of the performance improvement of the training process.

**Figure 6:** Average accuracy of task classification.

**Figure 7:** Accuracy of mental recovery in rock climbing sports without transcranial electrical stimulation.

**Figure 8:** Accuracy of psychological recovery in rock climbing with transcranial electrical stimulation.

**Table 1:** Advantages and disadvantages of different feature extraction methods.

Feature extraction method	Advantages	Disadvantages
Power spectrum analysis method	Simple algorithm, easy to operate	Low resolution, inability to display brain telecommunication nonlinear information of the number
Wavelet transform	Multiple resolutions for more detailed characterize the signal	Inflexible algorithm
Sample entropy method	Stable algorithm, low computational effort	Cannot express the time-frequency characteristics of the signal
Common spatial pattern method	Good performance in feature extraction for binary classification	Requires multiple leads for analysis and is susceptible to noise interference

**Table 2:** Experimental parameter setting.

Parameter name	Parameter value
Initial learning rate	0.002
Optimizer	Adam
Initial momentum	0.5
Batch size	30
Maximum number of training sessions	40

**Table 3:** Accuracy of subjects' psychological recovery from rock climbing exercise.

	Before stimulation	After pseudoarousal	After tACS	After tDCS
Subject 1	91.25	93.21	98.75	96.88
Subject 2	83.83	85.84	92.50	97.50
Subject 3	74.68	76.25	86.25	80.00
Subject 4	85.00	85.00	89.74	90.06
Subject 5	82.49	85.00	80.00	86.25
Subject 6	77.50	78.64	85.05	82.68
Subject 7	77.61	71.25	81.27	87.49
Subject 8	77.49	77.50	75.11	81.27
Subject 9	88.77	91.28	94.93	96.31
Mean ± standard deviation	82.07 ± 5.67	82.66 ± 7.25	87.07 ± 7.63	88.71 + 6.88

## Data Availability

The datasets used during the current study are available from the corresponding author on reasonable request.
